# Never-in-Mitosis A-Related Kinase 8 (NEK8) Regulates Adipogenesis, Glucose Homeostasis, and Obesity

**DOI:** 10.1155/2022/1947067

**Published:** 2022-11-30

**Authors:** Yan-Jun Wang, Ying Zhao, Yun-Wei Sun, Yan Chen

**Affiliations:** Department of Endocrinology, The Second Hospital of Jilin University, Changchun 130041, China

## Abstract

**Background:**

Adipogenesis is a complex biological process and the leading main cause of obesity. We evaluated the role of never-in-mitosis A-related kinase 8 (NEK8) in adipocyte development and insulin sensitivity in the present study.

**Methods:**

NEK8 expression was manipulated using a specific shRNA or the NEK8-full-length expressing recombinant plasmids. The interaction between NEK8 and Tafazzin (TAZ, an oncogenic transcriptional regulator) was examined by Co-immunoprecipitation (Co-IP) and confocal immunofluorescence staining. Western blot assay was performed to determine the protein expression. The *in vivo* role of NEK8 was explored in a mouse model of high-fat diet- (HFD-) induced insulin resistance.

**Results:**

During adipogenesis, the expression of NEK8 was elevated while TAZ was downregulated. Overexpression of NEK8 promoted lipid accumulation and expression of markers for adipocyte differentiation. Mechanically, NEK8 interacted with TAZ and suppressed its expression in adipocytes. Functionally, lentiviral-mediated NEK8 inhibition ameliorates HFD-induced insulin resistance in adipocytes.

**Conclusion:**

These findings suggest that NEK8 plays a critical role in adipocyte proliferation, providing novel insight into the link between NEK8 and type 2 diabetes- (T2DM-) related obesity.

## 1. Background

Type 2 diabetes (T2DM) has reached epidemic proportions and is the ninth major cause of death. T2DM is a complex, multifactorial disorder driven by genetic and environmental risk factors. Moreover, T2DM is a major risk factor for developing cardiovascular diseases [1–3]. Numerous studies have proven that adipose tissue is a subtle endocrine organ and plays an essential role in energy homeostasis. The abnormal function of adipocytes is closely related to lipid deposition, increased adipose tissue mass, and insulin resistance [4, 5]. Therefore, investigating the underlying mechanisms of adipogenesis may shed light on therapeutic strategies against T2DM.

Never-in-mitosis A-related kinase 8 (NEK8), also called NPHP9, is a member of the serine/threonine-protein kinase family and plays a critical role in cell cycle progression, primary cilia disassembly, and DNA damage response [6]. In addition, RNA interference-mediated NEK8 knockdown delayed gastric cancer cell proliferation, colony formation, and migration by interacting with von-Hippel-Lindau tumor suppressor protein (pVHL) [7]. It has been proposed that NPHP-associated disease mechanisms are achieved by regulating Wnt, Sonic hedgehog, and Hippo pathways [8, 9]. A previous study reported that NEK8 leads to nuclear translocation and activation of Tafazzin (TAZ, an oncogenic transcriptional regulator), thereby accelerating TAZ-mediated tumorigenesis [10]. In addition, TAZ was found to associate and to regulate obesity, and studies showed that mice that are knockdown of TAZ are protected from diet-induced obesity [11, 12]. Meanwhile, loss of NEK8 leads to abnormal organ development, and this effect was dependent on the activation of the Hippo pathway member TAZ [13]. However, the expression pattern and functional relevance of NEK8 and TAZ in adipogenesis remain unknown.

In the present study, we first investigated the functional role of NEK8 in adipocyte function and its association with TAZ using an *in vivo* model of HFD-induced type 2 diabetes in C57/BL6 mice. This research would be helpful for understanding the mechanisms of NEK8 in type 2 diabetes- (T2DM-) related obesity.

## 2. Materials and Methods

### 2.1. Cell Culture

3T3-L1 cells and HEK293T cells were purchased from the American Type Culture Collection (ATCC, Manassas, VA, USA) and maintained in DMEM (Gibco, Carlsbad, CA, USA) supplemented with 10% fetal bovine serum (FBS, Gibco, Carlsbad, CA, USA). Cells were maintained in a humidified incubator with 5% CO_2_ at 37°C. For standard induction of adipocyte differentiation, the confluent 3T3-L1 cells were incubated with the differentiation media (plus 0.5 mM isobutylmethyl xanthine, 1 *μ*M dexamethasone, and 10 *μ*g/mL insulin) for 48 hours. The differentiation pattern was studied both by observing the morphological changes and by estimating oil droplet accumulation in the cells. The differentiated adipocytes in culture after 4–10 days were taken for oil red O staining and to evaluate for its ability to glucose uptake.

### 2.2. Transfections

Transfections of plasmid DNA or shRNA were performed using the Lipofectamine 2000 (Thermo Fisher Scientific, Inc., Waltham, MA, USA) according to the manufacturer's instructions. The NEK8 overexpression was conducted by constructing the full-length NEK8 sequences into cells via pEX-2 plasmids (GenePharma, Shanghai, China). The pLKO lentiviral shRNA specific for NEK8 was obtained from Addgene (Cambridge, MA, USA), and a negative control (NC) shRNA was obtained from Genechem (Shanghai, P.R. China).

### 2.3. Quantitative Real-Time PCR (qRT-PCR)

Total RNAs were isolated from cells using Trizol Reagent (Invitrogen, USA) and reversely transcribed into cDNA using QuantiTect Reverse Transcription Kit (Qiagen). The relative expression of genes was measured by qRT-PCR. The assay was performed using SYBR Premix Ex Taq^TM^ (Takara, Otsu, Japan) on an Applied Biosystems 7500 Real Time machine (Applied Biosystems, Foster City, CA, US). The following primers used were NEK8-F, 5′-GTTCACCGCTTGCTTGACAG-3′, NEK8-R, and 5′-GGCTTCTACAATGGTGGGCT-3′; TAZ-F, 5′-ATGGGTAGGAATTGGACGGC-3′, TAZ-R, and 5′-GCTCAAGCACAGGGAGT GTA-3′; *β*-actin F, 5′-ACCCTAAGGCCAACCGTGAAA-3′, *β*-actin-R, and 5′-ATGGCGTGAGGGAGAG CATA-3′.

### 2.4. Western Blot

Total protein lysates were extracted from cells transfected with shRNA and overexpression plasmid. Briefly, the cells were washed with PBS, lysed with a mammalian lysis buffer (50 mM Tris-Cl, pH 8.0, 150 mM NaCl, 1 mM EDTA, 1% Nonidet P-40, and 0.4 mM phenylmethylsulfonyl fluoride (PMSF)) and sonicated, then denatured by incubation for 5 min at 95°C in a sample buffer (2% SDS, 10% glycerol, 60 mM Tris (pH 6.8), 5% *β*-mercaptoethanol, and 0.01% bromophenol blue). After that, the samples were subjected to 4-20% sodium dodecyl sulfate-polyacrylamide gel electrophoresis (SDS-PAGE) for fractionation and then transferred to polyvinylidene difluoride (PVDF) membranes and were blocked in skimmed milk at room temperature for 1 hour. Membranes were incubated with the primary antibodies (including anti-NEK8, TAZ, Pref-1, Adiponectin, PPAR*γ*, FABP4, and PEPCK antibodies overnight at 4°C. After being washed three times with PBST buffer, the membranes were incubated with secondary antibodies conjugated with horseradish peroxidase for 1 hour at room temperature. Protein bands were detected by enhanced chemiluminescence (ECL) method. Antibodies were used, including rabbit anti-NEK8 antibody (1 : 1000, Abcepta), rabbit anti-TAZ antibody (1 : 1000, Abcam), mouse anti- Pref-1 antibody (1 : 500, Bio-Techne), mouse anti-Adiponectin antibody (1 : 1000, Abcam), rabbit anti-PPAR*γ* antibody (1 : 2000, cell signaling), rabbit anti-FABP4 antibody (1 : 1000, Abcam), and rabbit anti-PEPCK antibody (1 : 1000, Sigma). Secondary antibodies included HRP-conjugated goat anti-rabbit IgG antibody and anti-mouse IgG antibody (1 : 2000, Jackson).

### 2.5. Immunoprecipitation

3T3-L1 cells were transiently transfected with the NEK8 overexpression plasmid with 0, 0.5, 1, and 2 *μ*g, and then incubated for an additional 48 hours. Then, 3T3-L1 cells were collected and lysed in RIPA lysis buffer (Yeasen, Shanghai) supplemented with protease inhibitor cocktail (Yeasen) for 30 min at 4°C, centrifuge at 8, 800 rpm for 10 min, and the supernatant was collected and divided into three 1.5 ml tube (one for input, one for IgG, and one for IP). Immunoprecipitation was conducted using antibodies against NEK8 or TAZ. Briefly, 1 *μ*g primary antibody against NEK8 or TAZ was added to 200 *μ*L cell lysates and incubated with rotation at 4°C for 2 h. Rabbit immunoglobulin G (IgG) was used as a negative control. Subsequently, proteins were precipitated with agarose A/G (Santa Cruz) and washed 5-6 times with RIPA lysis buffer. Immunoprecipitates and input were subjected to run SDS-PAGE, the next step same as western blot assay.

### 2.6. Immunofluorescence

The expression of NEK8 and TAZ were measured through immunofluorescent staining method. Briefly, cells were fixed for 15 minutes with 4% paraformaldehyde, permeabilized with 0.1% Triton X-100, blocked with blocking buffer, and incubated with indicated primary and secondary antibodies. Finally, the nuclei of the cells were stained and mounted with DAPI-Fluor mount reagent. All images were observed by a Nikon A1 microscope (Nikon, Japan).

### 2.7. Insulin-Stimulated 2-Deoxyglucose Uptake

3T3-L1 cells were incubated in FBS- and glucose-free DMEM at 37°C for 2 h and subsequently stimulated with 10 *μ*g/mL insulin for 30 min. Then, the glucose uptake and lactate product were measured using the Glucose Uptake Assay Kit (ab136955) from Abcam (Shanghai, China) according to the manufacturer's instructions.

### 2.8. Animals and Groups

The study protocol was approved by the Animal Care and Ethics Committee of College of Veterinary Medicine of Jilin University (Changchun, China). A total of 24 male C57BL/6 mice (age, 6 to 8 weeks; weight, 32–36 g) were purchased from Shanghai SLAC Laboratory Animal Co., Ltd. (Shanghai, China). Mice were housed with a 12 h light-dark cycle at 23 ± 2°C and 70% humidity, with free access to water and food. Mice were randomly divided into 4 groups, and each group contains six animals and was kept on normal chow or HFD. We observed that after 4 weeks of HFD feeding, the mice will produce a significant increase in body weight, basal/fasting plasma glucose, insulin, basal triglyceride, and total cholesterol levels. Thus, the mice were injected with lentiviruses carrying NEK8 shRNA through the tail vein after 4 weeks of HFD feeding. Body weight was measured weekly. The epididymal white adipose tissue (eWAT) was collected immediately after mice sacrificed at 6 weeks, frozen in liquid nitrogen, and stored at -80°C for later analysis.

### 2.9. Metabolic Experiments

Intraperitoneal glucose tolerance test (IPGTT) and intraperitoneal insulin tolerance test (ITT) were performed to examine the metabolic manifestation. For IPGTT, glucose at 2 g/kg was intraperitoneally administered, and blood glucose was measured at 0, 15, 30, 60, 90, and 120 min. For ITT, insulin at 0.75 IU/kg was intraperitoneally injected, and blood glucose was measured at 0, 15, 30, 60, 90, and 120 min.

### 2.10. Statistical Analysis

Experimental data were presented as mean ± standard deviation (SD) and analyzed using SPSS 20.0 software (IBM, Almond, NY, USA). Student's *t*-test was used for comparison between two groups. For more than two groups, mean values were compared using one-way ANOVA followed by the Dunnett's posttest. Values of *P* < 0.05 were considered statistically significant.

## 3. Results

### 3.1. NEK8 Was Gradually Upregulated during Adipocyte Differentiation in 3T3-L1 Cells

Representative images of differentiating 3T3-L1 adipocytes were observed by optical microscopic observation and oil red O staining. Before differentiation, the cells displayed a fibroblast phenotype; whereas, after 4 days of the differentiation process, the cells were more rounded and compact. On day 10, small droplets of triglycerides were visible in the periphery of the cells. In addition, cells were treated with oil red O to confirm triglyceride accumulation (Figure 1(a)).

The mRNA expression pattern of NEK8 during adipogenesis in 3T3-L1 cells was evaluated by qRT-PCR, and our data showed that NEK8 mRNA level was significantly increased at the time of induction on day 4 and day 10 (Figure 1(b)). A previous study demonstrated that TAZ is a negative regulator of PPAR*γ* activity in adipocytes [14], and our data showed TAZ was gradually suppressed during adipogenesis in 3T3-L1 cells (Figure 1(c)). Moreover, the western blot assay was performed to detect the protein expression level of NEK8, TAZ, as shown in Figure 1(d). Our western blot data confirmed that protein expression variation of NEK8 and TAZ paralleled mRNA levels during adipogenesis in 3T3-L1 cells (Figure 1(d)). Further, the adiponectin and PPAR were increased, and Pref-1 was decreased during adipogenesis in 3T3-L1 cells (Figure 1(d)).

### 3.2. NEK8 Physically Associated with TAZ

In addition, we evaluated the effects of TAZ on the expression of NEK8. Western blot assay showed that NEK8 overexpression represses TAZ in a dose-dependent manner in 3T3-L1 cells (Figure 2(a)). Collectively, these data suggested that NEK8 and TAZ are involved during adipogenesis. Given that NEK8 serves as a regulator of TAZ, we performed Co-immunoprecipitation (Co-IP) assays to explore whether NEK8 can interact with TAZ. We immunoprecipitated the proteins by using an anti-NEK8 (Figure 2(b)) and anti-TAZ (Figure 2(c)) antibody in 3T3-L1 cells. Co-IP assays showed that TAZ was detected in the samples immunoprecipitated by the anti-NEK8 antibody but not in those immunoprecipitated by IgG (Figure 2(b)), while the NEK8 was detected in the samples immunoprecipitated by the anti-TAZ antibody (Figure 2(c)). Furthermore, we explored whether NEK8 and TAZ are colocalized by confocal immunofluorescence microscopy. Consequently, both NEK8 and TAZ were localized in the cytoplasm in 3T3-L1 and HEK293T cells. The merged images revealed the clear colocalization of the two proteins (Figure 2(d)). These results confirm the specific interaction of NEK8 and TAZ.

### 3.3. NEK8 Promotes Adipogenesis in 3T3-L1 Cells

To unequivocally prove an effect of NEK8 on adipogenesis, the markers of terminally differentiated adipocytes [15](which enhance 3T3-L1 fibroblast proliferation and accelerate adipocyte differentiation) and undifferentiated preadipocytes [16](which is highly expressed in 3T3-L1 cells but is extinguished during adipocyte differentiation) were determined by western blot, as shown in Figure 3(a), and the adiponectin and PPAR*γ* were increased, and TAZ and Pref-1 were decreased in NEK8-overexpressed 3T3-L1 cells. In contrast, the adiponectin and PPAR*γ* were decreased, and TAZ and Pref-1 were increased in NEK8-silenced 3 T3-L1 cells. Moreover, our data revealed that knockdown of NEK8 significantly suppressed the accumulation of intracellular lipids, as evidenced by oil red O staining, while overexpression of NEK8 enhanced the lipid deposition (Figure 3(b)). Furthermore, we assessed the effects of NEK8 on the expression of markers for adipocyte differentiation. Western blot assay showed that the protein expression levels of PPAR*γ* and the target genes FABP4 and PEPCK were significantly decreased following NEK8 silencing, while overexpression of NEK8 significantly promoted these proteins expression (Figure 3(a)). In addition, insulin-stimulated glucose uptake was sensitized in 3T3-L1 adipocytes transfected with NEK8, whereas knockdown of NEK8 led to glucose tolerance (Figures 3(c) and 3(d)). These results suggest that NEK8 acts as a regulator of adipocyte differentiation and function.

### 3.4. Inhibition of NEK8 Improved Insulin Sensitivity in HFD-Fed Mice

We further explored the functional significance of NEK8 using HFD-fed mice. The body weight of mice injected with shNEK8 was obviously decreased compared to HFD mice and shNC + HFD mice (*P* < 0.001) (Figure 4(a)). To further evaluate the effect of NEK8 inhibition on insulin sensitivity, IPGTT and ITT assays were performed in this research. As shown, NEK8-silienced HFD mice have the lowest glucose levels during IPGTT and ITT compared to HFD and shNC + HFD mice (*P* < 0.001). Moreover, we found the increased expression of NEK8, and PPAR*γ* in the epididymal white adipose tissue was significantly decreased in NEK8-inhibited HFD mice (Figure 4(d)). These *in vivo* data confirmed that NEK8 affects glucose homeostasis under pathological conditions.

## 4. Discussion

The NIMA-related kinase (NEK) family of serine/threonine kinases is critical regulators of cell proliferation, primary cilia disassembly, and DNA damage response [17], and one family member is NEK8, which has a broad tissue distribution and was initially discovered in a juvenile cystic kidney mouse [14, 18]. NEK8 is a critical component of the DNA damage response that links replication stress with cystic kidney disorders [19]. Additionally, NEK8 has been identified as a tumor-associated gene that promotes cancer cell proliferation, colony formation, and migration [20].

In the present study, we explored the regulatory role of NEK8 in 3T3-L1 adipocyte differentiation and the underlying mechanism. We observed a significant elevation of NEK8 during adipogenesis (Figure 1). Functionally, knockdown of NEK8 significantly suppressed lipid accumulation and adipogenic gene expressions, such as PPAR*γ*, FABP4, and PEPCK (Figure 3(a)), leading to inhibition lipid deposition (Figure 3(b)). Moreover, silencing of NEK8 also inhibited insulin-stimulated glucose uptake *in vitro* (Figures 3(c) and 3(d)), which supported *in vivo* experiments. Collectively, these results suggest that NEK8 acts as a regulator of adipocyte differentiation and function.

Furthermore, we identified that TAZ was physically associated with NEK8 (Figure 2), and TAZ is a negative regulator of PPAR*γ* activity in adipocytes [21]. Based on these findings, there was no doubt that NEK8 possesses a positive regulatory on adipocyte differentiation by interacting and transcriptionally repressing TAZ, thereby regulating glucose homeostasis and insulin sensitivity.

The Hippo pathway is an important hub coordinating cell proliferation and differentiation to regulate tissue growth [22]. TAZ, also called WWTR1, is a critical effector of this pathway and regulates cell proliferation, survival, and differentiation. A large amount of evidence has confirmed the functional relevance of TAZ during adipogenesis [23, 24]. A previous study demonstrated that TAZ suppression increased the lipid deposits and adipogenic gene expression in 3T3-L1 cells [25]. Recently, knockdown of TAZ has been reported to improve glucose tolerance and insulin sensitivity in obese mice [21]. Our data showed that overexpression of NEK8 significantly suppressed TAZ expression in the present study (Figure 2(a)). Moreover, the interaction of NEK8 and TAZ was measured by Co-IP and confocal immunofluorescence approach, and our data demonstrate NEK8 is physically associated with TAZ (Figures 2(b)–2(d)), indicating that NEK8 interacted with TAZ to regulate adipocyte differentiation and functions. Nevertheless, the precise mechanism by which NEK8 regulates TAZ and its downstream pathway needs further investigation.

The *in vivo* research of NEK8 knockdown was performed in HFD-fed mice, as shown in Figure 4, and the bodyweight of mice injected with shNEK8 was decreased compared to HFD mice and shNC + HFD mice. In addition, we evaluated the effect of NEK8 inhibition on insulin sensitivity, and our data showed NEK8-inhibited HFD mice have the lowest glucose levels during IPGTT and ITT (Figures 4(a)–4(c)).

In conclusion, our study identified that NEK8 is physically associated with TAZ and promotes adipocyte differentiation. These findings provide a novel insight into the link between NEK8 and metabolic disorders.

## Figures and Tables

**Figure 1:** NEK8 was gradually upregulated during adipocyte differentiation in 3T3-L1 cells. (a) 3T3-L1 preadipocytes in FBS-containing medium were treated with 1 *μ*M dexamethasone, and the images of 3T3-L1 were observed under optical microscopy and visualized by oil red O staining. The mRNA levels of (b) NEK8 and (c) TAZ were examined by real time PCR, and the protein levels of NEK8, TAZ, adiponectin, Pref-1, and PPAR*γ* were examined by western blot. (d) *β*-Actin was used as a loading control. The data are represented as mean values ± SD from three independent experiments in triplicate, ^∗^*P* < 0.05, and ^∗∗^*P* < 0.01.

**Figure 2:** NEK8 physically associated with TAZ. (a) 3T3-L1 cells were transiently transfected with the NEK8 overexpression plasmid with 0, 0.5, 1, and 2 *μ*g and then incubated for an additional 48 hours, and the cell lysates were collected to determine the NEK8 and TAZ level by western blot assay and *β*-actin as a loading control. (b, c) Co-immunoprecipitation (Co-IP) was conducted to detect the interaction between NEK8 and TAZ, and IgG was used as a control. (d) Confocal immunofluorescence staining was used to detect the colocalization of NEK8 and TAZ.

**Figure 3:** NEK8 promotes the adipogenesis in 3T3-L1 cells. 3T3-L1 cells were transiently transfected with the NEK8 shRNA and overexpression plasmids and then incubated for 4 days. (a)The protein levels of NEK8, TAZ, adiponectin, Pref-1, PPAR*γ*, FABP4, and PEPCK were examined by western blot and *β*-actin as a loading control. (b) Representative images of differentiating 3T3-L1 adipocytes after oil red O staining. (c, d)The insulin-stimulated glucose uptake was determined in 3T3-L1 cells under NEK8 silenced or overexpressed. The data are represented as mean values ± SD from three independent experiments in triplicate, ^∗^*P* < 0.05, and ^∗∗^*P* < 0.01.

**Figure 4:** Inhibition of NEK8 improved insulin sensitivity *in vivo.* (a) Body weight, (b) IPTGG, (c) and ITT in normal, HFD-fed mice injected with shNEK8 or shNC (*n* = 6). (d) Protein expressions of NEK8 and PPAR*γ* in the epididymal white adipose tissue were examined by western blot. The data are represented as mean values ± SD from three independent experiments in triplicate,^∗^*P* < 0.05, ^∗∗^*P* < 0.01, and ^∗∗∗^*P* < 0.001.

## Data Availability

The datasets used and/or analyzed during the current study are available from the corresponding author on reasonable request.
